# Correlation of Computed Tomographic Angiography in Patients Undergoing Coronary Artery Bypass Grafting and Effect of Standardized Rehabilitation Nursing

**DOI:** 10.1155/2022/6184061

**Published:** 2022-06-14

**Authors:** Mingming Liu

**Affiliations:** Department of Cardiovascular Surgery, The First Affiliated Hospital of Harbin Medical University, Harbin 150000, China

## Abstract

This study aimed to explore the clinical application of computed tomographic angiography (CTA) and standardized rehabilitation nursing in patients with coronary artery bypass grafting (CABG). CTA image was segmented by reconstruction algorithm and finally assembled into a whole image. Three-dimensional reconstruction of the coronary artery was then performed. 52 patients were selected as the research objects, and standardized rehabilitation nursing was carried out after surgery to analyze the vascular lesion rate of arterial bridge and venous bridge and compare their nursing satisfaction. The results showed that the CTA images were clearer after reconstruction. The number of male patients with venous and arterial lesions was significantly higher than that of the female patients, and the difference between the two groups was obvious (*P* < 0.05). The number of patients combining with risk factors and LIMA bridge vessels was 0 in grade 3 patients, accounted for the highest proportion (16.67%) in the grade 1 patients, and was 2 in the grade 2 patients (accounting for 4.17%). The satisfaction of patients who received standardized nursing was 97.25%, that of patients who received conventional nursing was 83.42%, and the difference was significant (*P* < 0.05). In conclusion, CTA images of patients' cardiac vessels can be clearly seen by using a block image reconstruction algorithm, which can realize clinical personalized treatment. In addition, patients were more satisfied with standardized rehabilitation nursing.

## 1. Introduction

Coronary atherosclerotic heart disease (coronary artery disease for short) is a kind of atherosclerotic heart disease, which is a common clinical disease [1]. Relevant data show that the death rate of coronary heart disease ranks second in the world, and there are about 11 million patients with coronary heart disease in China. The main treatments for CHD are lifestyle changes, medication, and surgery [2]. Coronary artery bypass grafting (CABG) is a kind of surgery to improve cardiac and myocardial blood supply to the heart by restoring or replacing the coronary artery obstruction. When the coronary arteries are less than 50%, it has little influence on blood flow, and drug treatment can have a satisfactory curative effect. However, if the stenosis reaches 75%, there will be significant obstruction of blood flow and angina symptoms, requiring stent surgery.

At present, invasive angiography (ICA) is the gold standard of CABG [3, 4]. At present, the development of noninvasive diagnostic methods such as electron beam computed tomography (CT) (EBCT), multislice spiral CT (MSCT), and magnetic resonance imaging (MRI) provides a variety of options for the diagnosis of clinical diseases. Computed tomographic angiography (CTA) is widely used in clinical practice, and powerful imaging treatment methods can clearly present the coronary arteries from various perspectives [5, 6]. The proximal and distal anastomosis of the bridging vessel, the bridging vessel, and the relationship between the titanium clip of the lateral branch of the internal mammary artery and the normal vessel wall can also be clamped by rotating [7]. CTA is a safe noninvasive coronary artery examination. The contrast agent is injected into the patient's body through the cubital vein at a delivery rate of 3–5 mL/s. Then, artificial intelligence software is used to control the contrast agent tracking technology and cardiac gating to clearly display the coronary arteries and their branches, as well as the movement of the heart chamber wall [8, 9]. Finding a reliable and noninvasive method to check the coronary arteries is the direction of clinical cardiology research. Spiral CT cardiac CTA scanning has been widely recognized by both doctors and patients in clinic for its advantages of low radiation damage, convenient examination, fast scanning speed, and low cost [10]. CTA examination can obtain the patency of one-stop coronary arteries and related indicators of cardiac function. The measurement results of cardiac function are highly consistent with echocardiography and MRI, and CTA examination has become a routine imaging examination method before and after CABG [11].

CHD is a chronic disease, and in addition to the need for good treatment and diagnosis methods, postoperative care also plays an important role in the prognosis of patients to improve the survival rate and quality of life of patients. Standardized rehabilitation nursing is one of the nursing methods that are used more and more concerned in clinical practice [12]. Some foreign scholars use standardized rehabilitation care to reduce the incidence of CHD by 50%. Research by domestic scholars has shown that standardized rehabilitation nursing can improve the comfort, satisfaction, and compliance of clinical treatment [13]. In summary, the standardized rehabilitation nursing has achieved good results in clinical work and has been widely promoted. However, the application of standardized rehabilitation care directly to the postoperative recovery of patients with CABG is less in clinical practice [14].

The iterative reconstruction algorithm is an image reconstruction technique, which can obtain diagnostic images under low scanning conditions. Although the iterative algorithm has a large amount of computation and takes a long time, it is still considered to be a better reconstruction method for incomplete projection and projection data with noise [15]. The iterative algorithm divides the whole process of the image into many times and improves the image processing step by step. In most low-dose scanning, the image processing parameters must be optimized to improve the image quality to the maximum extent. The algorithm and various noise reduction technologies can achieve the role of smoothing the image. The optimization of the CT reconstruction algorithm can greatly reduce the noise value on the image and improve the signal-to-noise ratio (SNR) by using the original CT data collected through repeated massive operations of mathematics and physics. Thus, the radiation dose of patients is reduced, the image quality is improved, and the spatial resolution and density resolution of the image are improved. Therefore, it is of great significance to explore the efficient CT reconstruction algorithm, make full use of the advantages of the algorithm, and flexibly apply it to clinical practice. At present, most of the reconstruction algorithms are applied to the processing of ultrasound images in China, but there are few studies that apply them to the processing of CTA images.

In this work, dual-source CT was used to perform coronary CTA examination to obtain preoperative and postoperative cardiac function indicators of patients with CABG, and the factors for improving cardiac function after imaging CABG were analyzed. The reconstruction algorithm was used to improve the image quality of low-dose CT reconstruction. Analytical reconstruction and statistical iterative reconstruction are the most commonly used methods for CT reconstruction. Compared with the analytic reconstruction algorithm, the iterative algorithm is more flexible in the calculation, and the original image can be reconstructed using only the projection data, so as to obtain more accurate treatment diagnosis results. It aimed to provide more comprehensive and detailed imaging information for patients with CABG and to deeply understand the combination of vascular morphological changes and hemodynamic changes. The characteristics of patients were analyzed from different perspectives to provide a reference for clinical treatment and nursing of patients with CABG.

## 2. Methods and Materials

### 2.1. Selection of Patients

Fifty-two patients who received CABG treatment in the hospital from January 2018 to January 2020 were selected as the research objects. There were 32 males and 20 females, aged 42–72 years old, with an average age of 61.31 ± 6.51 years old. All the patients had complete clinical data and follow-up data, with a total of 87 bridging vessels, of which 47 were arterial bridges and 40 were venous bridges. This study had been approved by the ethics committee of the hospital, and all relevant patients signed the informed consent forms.

Inclusion criteria were as follows: patients who were clinically diagnosed with CHD; patients with complete clinical data; patients who could cooperate with medical workers independently; patients who had not interrupted the treatment in this hospital; and patients who met the treatment indications.

Exclusion criteria were as follows: patients with severe cardiac and renal disease and allergy to iodinated contrast media must be excluded; patients with communication disorder; patients with poor treatment compliance; patients with mental diseases; patients who stopped treatment due to multiple reasons; and patients with arrhythmia, such as those who cannot control the heart rate below 70 times through drugs.

### 2.2. Reconstruction Algorithm

The general filtering backprojection reconstruction algorithm is mainly aimed at the projected data reconstruction of the whole image, the reconstruction of the image requires a very high resolution, and the corresponding reconstruction time will be doubled. The block image reconstruction algorithm divides projection space and image into blocks. After each image is calculated, it is integrated into the whole image. The reconstructed image does not need to be realized on an expensive special machine but needs to be simultaneously reconstructed in different pieces on a computer. Single block image reconstruction consumes less resources than the whole image reconstruction, which can reduce the radiation damage caused by X-ray to the human body.

Function *F* (*q*, Φ) was the value of a physical quantity at the coordinate (*q*, Φ). The position of the projection ray at point *F* (*q*, Φ) was represented by (*m*, *θ*), which was expressed as *f*(*x*, *y*) in the rectangular coordinate system. −*M* ≤ *m* ≤ *M*; −*M* ≤ *m*' ≤ ; 0 ≤ *φ* ≤ *π*; −*E* ≤ *x* ≤ *E*; −*E* ≤ *y* ≤ *E*.

*θ* was the segmentation parameter, *P* referred to the parameter *m*, *I* was the parameter *x*, and *y* represented the Cartesian coordinate system representing the image space. The rectangular coordinate system of *θ* was mouse projection space, *D* represented parameter *m*, and the rectangular coordinate system of *θ* represented filtering projection space.

(1) $$\begin{array}{c} P=\left\{\left(m,\theta \right)\right\}-M\leq m\leq M,0\leq \theta \leq \pi ,\\ D=\left\{\left(m^{\prime },\theta \right)\right\}-M\leq m^{\prime }\leq M,0\leq \theta \leq \pi ,\\ I=\left\{\left(x,y\right)-W\leq m\leq W,-W\leq y\leq W\right\}=\left\{\left(q,\Phi \right)|-W\leq q\text{cos}\Phi \leq W,-W\leq q\text{sin}\Phi \leq W\right\}. \end{array}$$

### 2.3. Algorithm Steps

Block filtering divides spatial parameters into *N* word blocks, meeting the following conditions:

(2) $$\begin{array}{c} \overset{N}{\underset{N=1}{\cup }}P_{N}=P,\\ P_{N}\cap P_{i}=0,\;\left(N\neq i\right), \end{array}$$

∀ (*m*, *θ*) *∈ P k*, then the (3) could be obtained

(3) $$\begin{array}{c} P_{d}\left(m,\theta \right)=P\left(m,\theta \right)*q\left(m\right). \end{array}$$

And then, *k* was obtained.

Filter projection data are assembled, and the obtained data are assembled into *D* in sequence, which satisfies the following equation:

(4) $$\begin{array}{c} D=\overset{N}{\underset{N=1}{\cup }}D_{N}. \end{array}$$

The back projection after blocking was segmented according to the parameters, *x* and *y* were segmented into *I*, satisfying *S* = *M* × *N*, and the word block was Is, which satisfied the following equation.

The set of projection position (*m*′, *θ*) of *Sj* through region *Ij* filter was determined according to the classifier.

The reconstructed image was assembled. It was assembled into *I* in the order of *x* and *y* according to the subblocks generated in the target space, and then, (5) was obtained.

(5) $$\begin{array}{c} I=\overset{J}{\underset{j=1}{\cup }}I_{j}. \end{array}$$

The specific flow chart for image processing was given in Figure 1.

### 2.4. The Index of Image Evaluation

The precision (Pre), Dice coefficient, and sensitivity [18] were used to evaluate. Equations (6) − (8) showed the calculations of these three indexes.

(6) $$\begin{array}{c} \text{Dice}=\frac{\left[2\left(\Omega \text{Seg}\cap \Omega Gr\right)\right]}{\left(\Omega \text{Seg}＋\Omega Gr\right)}=\frac{2\text{TP}}{\left(2\text{TP}＋\text{FP}＋\text{FN}\right)}, \end{array}$$

(7) $$\begin{array}{c} \text{Precision}=\frac{\left(\Omega \text{Seg}\cap \Omega Gr\right)}{\Omega \text{Seg}}=\frac{\text{TP}}{\left(\text{TP}＋\text{FP}\right)}, \end{array}$$

(8) $$\begin{array}{c} \text{Sensitivity}=\frac{\left(\Omega \text{Seg}\cap \Omega Gr\right)}{\Omega Gr}=\frac{\text{TP}}{\left(\text{TP}＋\text{FN}\right)}. \end{array}$$

### 2.5. CTA Examination and Its Precautions

Precautions before CTA examination: 64-row spectral CT was used. Firstly, 4 hours before the examination, the patient was not allowed to eat solid food but could drink water. Secondly, if the patient was in excessive tension, it could take oral tranquilizers half an hour before the examination. Thirdly, patients were required to not do any exercise but sit in the examination room in advance to stabilize the heart rate. Fourthly, caffeinated beverages were not accepted within 12 hours before the examination. Finally, the doctor gave some drug treatment and breathing training guidance according to the specific situation of the patient.

CTA scanning: all patients were examined using a DSCT scanner in a supine position, positioning images from the thoracic entrance to the heart septum. The heart calcification score of patients was scanned. The scanning range was 10–15 mm below the organ bifurcation to the diaphragmatic surface of the heart. The scanning parameters were set as follows: tube voltage was 120 kV, the tube current was 100 mKs, and the scanning time was 7–11 s. For enhanced scanning, a 10 mm layer from the upper abdomen of the left trunk opening to the heart surface was selected, the collimation was 32 × 0.6 mm, the voltage was 120 kV, the rotating speed of the tube ball was 0.27 s/ROT, the pitch was automatically matched with the psychology by 0.2–0.43, the scanning time was 5–12 s, and the breath-holding scan was performed. The speed of syringe injection was 4.5–5.0 mL/s, the injection volume was 370 mgI/mL, the dosage of iodine contrast agent was 75–80 mL, and then, 50 mL of normal saline was injected at the same flow rate. After image reconstruction, the thickness was 0.75 mm, and the reconstruction interval was 0.5 mm. The contrast agent tracer method was selected to start the scanning, and the region of interest (ROI) was selected at the aortic root level with a trigger threshold of 100HU. After the scan, the image was processed, the calcification score of the patient was analyzed in-depth, and the image surface reconstruction and maximum projection were compared.

### 2.6. Image Processing

After the scan, the image was processed, the calcification score of the patient was analyzed in-depth, and the image surface reconstruction and maximum projection were compared. Data of CTA examination were reconstructed after using R-R interval 0–100% of the time reconstruction. The layer thickness and apart of the reconstructed image were 1.5 mm and 0.7 mm, respectively. The images were transmitted to the MMWP workstation and analyzed by circulation function analysis software. The position of the four-chamber heart, the long axis position, and the short axis position of the left ventricle were selected, and each cardiac cycle was played back. The software was used to delineate the boundaries of the internal and external modes of left ventricular muscle in systolic and diastolic stages, and the software was used to calculate the left ventricular end-systolic volume (LVESV), left ventricular ejection fraction (LVEF), left ventricular end-diastolic volume (LVEDV), and left ventricular stroke volume (LVSV) automatically.

### 2.7. Assessment of the Severity of Coronary Arteries Stenosis

The classification method to determine the severity of coronary artery stenosis was based on the classification standard recommended by the Cardiology Branch of Chinese Medical Association. The internationally accepted diameter method was used to evaluate the degree of stenosis. Clinically, it was divided into the severe stenosis group (stenosis >70%) and the moderate stenosis group (stenosis >50% and ≤70%). The degree of vascular stenosis was represented by *W*, the diameter of the normal proximal vascular stenosis was *d*, the diameter of the stenosis was *d1*, and the proximal vascular stenosis was *d*2. The degree of vascular stenosis *W* was calculated by the following equation:

(9) $$\begin{array}{c} W=\frac{d-d1}{d2}\times 100\%. \end{array}$$

Vascular lesions were grouped according to Fitz Gibbon standard [16], and the stenosis grades were shown in Table 1.

### 2.8. Standardized Nursing

Patients received standardized nursing after surgery. Nursing staff should take psychological and physical nursing, communicate with patients' families, encourage patients to speak out their doubts, and take psychological and nursing assessments on patients.

### 2.9. Evaluation of Nursing Satisfaction

The nursing results were compared with the routine nursing satisfaction of 40 patients. The contents of the investigation of nursing satisfaction included service attitude, psychological nursing, nursing initiative, health education, and professional skills. There are 1–4 points for each item, with a minimum of 25 points and a total of 100 points. It was deemed as very satisfied when the score was above 86, as satisfied when the score was 71–85, as fair when it was 50–70, and as not satisfied when it was below 50. Nursing satisfaction = (very satisfied + satisfied)/total number of cases × 100%.

### 2.10. Observation Indicators

The main observation indicators were as follows: nursing satisfaction; algorithm performance evaluation indicators such as precision (Pre), Dice coefficient, and sensitivity; lesion rate of arterial bridge; occurrence of diabetes, hypertension, and hyperlipidemia; and LIMA bridge vascular classification.

### 2.11. Statistical Analysis

SPSS19.0 statistical software was used for data processing in this work. The measurement data conforming to normal distribution were expressed as mean ± standard deviation (*x*‾ ± *s*), and or otherwise, they were expressed as frequency or percentage (%). The difference was statistically significant with *P* < 0.05 and insignificant otherwise.

## 3. Results and Analysis

### 3.1. Image Reconstruction by Block Algorithm

The internationally used Shepp-Logan head illusion (Phantom) and simulation program were adopted, and the size of the image reconstructed by the block algorithm was 256 × 256. The simulation was taken using a parallel beam, and 360 projections were made within 180 degrees of scanning. The distance between projection elements was the same as that between pixels (Figure 2).

### 3.2. Comparison of Algorithmic Reconstruction Effects

The comparison results of the iterative reconstruction algorithm and the traditional algorithm reconstruction effect were shown in Figure 3. It revealed that the performance of the iterative reconstruction algorithm was significantly better than that of the traditional algorithm (*P* < 0.05).

### 3.3. CTA Examination Results

In Figure 4, the figure on the left was the case result of the examination of patients, and the figure on the right was the case proportion result. Among the 52 patients, there were 5 cases without tube wall stenosis, accounting for 9.62%, 11 cases with mild stenosis (21.15%), 24 cases of moderate stenosis (46.15%), 9 cases of severe stenosis (17.31%), and 3 cases of complete occlusion (5.77%).

### 3.4. Analysis of Images

Figure 5 shows the images of 61-year-old men with a heart rate of 50 BPM and exertional chest pain for more than 10 years, which could attack after going 2–3 floors. There was a narrow stent in coronary angiography. No obvious abnormalities were observed in the carotid artery. After the descending stent implantation before CTA coronary artery examination, the stent was unobstructed, and no obvious plaque or stenosis was observed in the corresponding vermilion vessels, indicating that the coronary arteries had minor vascular lesions. No heart cavity size structure was observed in the cardiac bypass, and the movement of the chamber wall and valve changed. The diet was light, and some exercise was ensured. The possible restenosis of stain was overdue, and lipid-lowering drugs can be stopped.

### 3.5. Analysis of Gender and Lesion Rate of Arterial Bridge

Among the 52 subjects, 32 were male and 20 were female. In arterial bridge LIMA, there were 7 male patients with lesions (the lesion rate was 13.46%) and 5 female patients with lesions (the lesion rate was 9.62%). There were 11 male patients (with a lesion rate of 21.15%) and 9 female patients (with a lesion rate of 17.31%) with venous bridge SV lesions. The number of men with venous disease and arterial disease were significantly higher than that of women, and there was a significant difference between the two groups (*P* < 0.05). The specific results were shown in Figure 6.

### 3.6. Analysis of Related Indicators of Patients

The clinical data of the patients were collected and analyzed. The “diabetes mellitus”, “hypertension”, and “hyperlipidemia” were undertaken as risk factors, and 48 patients were included in the standard classification. They were grouped according to the composite factor of resting vascular lesions, and the results were shown in Figure 7. The number of patients combining with risk factors and LIMA bridge vessels was 0 in grade 3 patients, accounted for the highest proportion (16.67%) in the grade 1 patients, and was 2 in the grade 2 patients (accounting for 4.17%).

As illustrated in Figure 8, the number of patients combining with risk factors and LIMA bridge vessels was 11 in grade 3 patients (accounting for 22.92%), 9 in grade 2 (accounting for 18.75%), and 1 in grade 3 patients (accounting for 2.08%).

### 3.7. Nursing Satisfaction Rate

In this work, 52 patients underwent standardized rehabilitation nursing after surgery, and their satisfaction was compared with the 40 patients who underwent conventional nursing during the same period. As demonstrated in Figure 9, the satisfaction rate in standardized nursing was 97.25%, while that in the conventional nursing was 83.42%, and the difference was significant (*P* < 0.05).

## 4. Discussion

Coronary arteries CTA imaging can well show the location and morphological structure of coronary arteries stents in patients after stent placement and the position of coronary arteries stents in patients after direct implantation. Among the 52 patients in this work, there were 5 cases without wall stenosis (accounting for 9.62%), 11 cases with mild stenosis (accounting for 21.15), 24 cases with moderate stenosis (accounting for 46.15%), 9 cases with severe stenosis (accounting for 17.31%), and 3 cases of complete occlusion (accounting for 5.77%). The proportion of patients with moderate stenosis was the highest. CTA imaging technology can accurately display myocardial bridges, and it also provides a basis for the clinical judgment of myocardial ischemia. CTA technology is another great progress in the diagnosis of coronary heart disease in recent years. Patients with coronary heart disease are asymptomatic in general. It can lead to acute myocardial infarction if insufficient attention is paid. CTA angiography has become a new trend in the diagnosis and screening of coronary heart disease. MSCT CTA plays an important role in the postoperative review of patients with coronary heart disease and the screening of underlying cardiac diseases in healthy people. Early detection and diagnosis of coronary arteries lesions can effectively prevent and reduce the incidence of myocardial infarction and sudden death myocardial infarction. Shah et al. (2019) [17] proved that coronary arteries CTA had general diagnostic accuracy and can provide more detailed anatomical information, and coronary arteries CTA can be applied to the diagnosis of heart transplant recipients. Ghekiere et al. (2017) [18] stated that CTA can be used for invasive assessment of cardiac and coronary arteries, but the image quality and diagnostic value in patient examinations were determined by both technical and patient-related factors.

As an important research branch of scientific computing visualization, the three-dimensional reconstruction of medical volume data needs to fit these discrete data on the computer and convert it into an image with an intuitive three-dimensional effect. It can use the characteristics of the human visual system to display the three-dimensionality of human organs, thereby improving some anatomical results information that cannot be obtained by traditional manual methods. Simulation experiments show that when the projection data are relatively complete, the filtered backprojection algorithm can obtain better reconstruction quality based on the parallel beam projection, and the fan beam projection data can be directly obtained by data rearrangement. Ru et al. (2021) [19] revealed that coronary arteries CTA was of great value in the detection of mounted arteries, which could accurately check the severity of coronary arteries stenosis and locate the stenotic lesions. In this work, the degree of stenosis of CABG patients was divided, and the proportion of patients in the second level was the highest. The postoperative satisfaction comparison found that the satisfaction on standardized nursing was 97.25%, and that on conventional nursing was 83.42%, with a significant difference between the two (*P* < 0.05).

## 5. Conclusion

In this work, the intelligent reconstruction algorithm was used to reconstruct the CTA imaging of CABG patients, which effectively improved the image feature extraction and classification efficiency of patients. The results of this work revealed that dual-source CT for coronary CTA can accurately identify the degree of coronary arteries stenosis in patients, and the patients' satisfaction reached 97.25% after standardized rehabilitation nursing. This study provided a reference and basis for the clinical diagnosis and treatment of CHD. In this work, image reconstruction took a long time, especially for high-resolution images. Therefore, how to shorten image reconstruction in future research is also a new research direction.

## Figures and Tables

**Figure 1:** Image processing flow chart.

**Figure 2:** Simulation effects of reconstructed images. (a) Projection data, (b) image algorithm, (c) image segmented by the algorithm, and (d) projection of the segmented image.

**Figure 3:** Comparison of ultrasonic image effect between the two groups. *∗* Compared with traditional algorithms, *P* < 0.05.

**Figure 4:** CTA examination results.

**Figure 5:** CTA images of a patient. The images from left to right were CTA cardiac image, coronary CTA image, coronary CTA image, and cervical vascular image, respectively.

**Figure 6:** Correlation of gender and vascular lesion rate. *∗* meant the difference was significant with *P* < 0.05.

**Figure 7:** Comprehensive risk factors and lesion rate of LIMA bridge.

**Figure 8:** Comprehensive risk factors and lesion rate of LV bridge.

**Figure 9:** Comparison of satisfaction. *∗* meant the difference was significant with *P* < 0.05.

**Table 1:** Group of the degree of vascular bridge lesion.

Degree	Vascular performance
*A*	Vascular was smooth without stenosis, and lumen patency was more than 50%
*B*	The vessels themselves were significantly narrowed, the remaining lumen was less than 50% in the oral cavity, and the bridge was not completely occluded
*O*	The bridge vessels were completely occluded without contrast

## Data Availability

The data used to support the findings of this study are available from the corresponding author upon request.
